The article "MicroRNA-133a suppresses colorectal cancer cell invasion by targeting Fascin1" was retracted in 2021. Reasons: duplicated images; signs of a paper mill.

# MicroRNA-133a suppresses colorectal cancer cell invasion by targeting Fascin1

**DOI:** 10.3892/ol.2014.2753

**Published:** 2014-12-01

**Authors:** KEYAN ZHENG, WEICHENG LIU, YE LIU, CONGQING JIANG, QUN QIAN

**Affiliations:** Department of Colorectal and Anal Surgery, Zhongnan Hospital of Wuhan University, Wuhan, Hubei 430071, P.R. China

**Keywords:** colorectal cancer, microRNA-133a, Fascin1, invasion

## Abstract

MicroRNAs (miRs) are a type of small non-coding RNA molecule that are involved in gene silencing and the regulation of cancer progression; miR-133a in particular has been implicated in colorectal cancer, although its specific role and underlying mechanism have yet to be determined. In the present study, the expression level of miR-133a was significantly downregulated in a number of colorectal cancer cell lines, as well as in colorectal cancer tissues compared with the normal adjacent tissues. Furthermore, the Fascin1 (FSCN1) gene was identified as a direct target of miR-133a, and the protein expression level of FSCN1 was negatively regulated by miR-133a in colorectal cancer cells. Additionally, restoration of miR-133a expression and downregulation of FSCN1 protein expression suppressed colorectal cancer cell invasion, while overexpression of FSCN1 reversed the inhibitory effect of miR-133a upregulation on colorectal cancer cell invasion. Thus, the present data indicates that miR-133a may at least partially suppress colorectal cancer cell invasion, possibly via the inhibition of FSCN1 expression. The present study highlights the important role of miR-133a in the progression of colorectal cancer.

## Introduction

Colorectal cancer is the third most common type of cancer and the third leading cause of cancer-related mortality among males and females in the United States (1), thus, it is important that effective therapeutic targets for colorectal cancer are identified.

The dysfunction of oncogenes or tumor suppressor genes is known to be involved in the development and progression of colorectal cancer (2). Recently, deregulation of microRNAs (miRNAs) that serve as tumor suppressors or oncogenes has been demonstrated to largely contribute to the development and progression of various types of cancer, including colorectal cancer (3,4). miRNAs are a class of 18- to 25-nucleotide non-coding RNAs that are able to induce mRNA degradation or inhibit protein translation by directly binding to the 3′-untranslated region (UTR) of their target mRNAs. By mediating the protein expression levels of their targets, miRNAs are involved in the regulation of cell survival, proliferation and migration, as well as cell cycle progression (5,6). Thus, the deregulation of various miRNAs has been identified as a critical factor in colorectal cancer (3,4). Among these miRNAs, miR-133a has been demonstrated to exhibit suppressive properties in numerous types of human malignancies, including non-small cell lung cancer (7), gastric cancer (8), osteosarcoma (9), esophageal squamous cell carcinoma (10), ovarian cancer (11) and colorectal cancer (12). However, the specific role of miR-133a in the regulation of colorectal cancer cell invasion is yet to be fully determined.

Fascin1 (FSCN1) is an actin-bundling protein and is well-established as an integral component of invadopodia, which stabilize actin bundles in invasive foot structures. Furthermore, it has been proposed that FSCN1 is involved in the regulation of cell motility and, thus, may be associated with cancer cell invasion (13,14). Recently, high expression levels of FSCN1 were reported to be associated with poor prognosis in patients with colorectal cancer, indicating that FSCN1 may act as an oncogene in colorectal cancer (15,16). However, the underlying mechanism by which FSCN1 mediates the progression of colorectal cancer is largely unknown.

The aim of the present study was to investigate the role of miR-133a in the regulation of colorectal cancer cell invasion *in vitro* and the underlying molecular mechanism of this process.

## Materials and methods

### Tissue specimens

The present study was approved by the Ethical Committee of Wuhan University (Wuhan, China). Colorectal cancer tissues (n=17), as well as the paired adjacent normal tissues, were obtained from the Department of Colorectal and Anal Surgery of Zhongnan Hospital, Wuhan University. Following surgical excision, the tissue samples were frozen in liquid nitrogen until required. Informed consent was obtained from each colorectal cancer patient.

### Cell culture

The human colorectal cancer cell lines, HT29, SW480 and SW620, as well as the normal intestinal epithelium cell line, NCM460, were purchased from the Cell Bank of Wuhan University and cultured in Dulbecco’s modified Eagle’s medium (DMEM) supplemented with 10% fetal bovine serum (FBS) in a 37°C atmosphere containing 5% CO_2_ .

### Reverse transcription-quantitative polymerase chain reaction (RT-qPCR) assay

Total RNA was extracted using TRIzol reagent (Life Technologies, Carlsbad, CA, USA), and a TaqMan^®^ miRNA Reverse Transcription kit (Life Technologies) was used to convert RNA into complementary DNA, according to the manufacturer’s instructions. RT-qPCR was performed using the All-in-One™ miRNA qRT-PCR detection kit (GeneCopoeia, Rockville, MD, USA) on an Applied Biosystems 7500 thermocycler (Life Technologies). The U6 gene was used as an internal reference and the relative expression was analyzed using the 2^−ΔΔCt^ method.

### Western blot analysis

Tissues and cells were solubilized in cold radioimmunoprecipitation assay lysis buffer, and the proteins were separated by 10% SDS-PAGE and transferred onto a polyvinylidene difluoride (PVDF) membrane. The PVDF membrane was incubated with phosphate-buffered saline containing 5% non-fat milk overnight at 4°C. Following incubation, the PVDF membrane was incubated with mouse monoclonal anti-FSCN1 (dilution, 1:400; cat. no. ab49815) and mouse monoclonal anti-GAPDH (dilution, 1:200; cat. no. ab8245) primary antibodies at room temperature for three hours, and then with rabbit anti-mouse monoclonal secondary antibodies (dilution, 1:20,000; cat. no. 175743) (Abcam, Cambridge, UK) at room temperature for one hour. Chemiluminescence was detected using an enhanced chemiluminescence kit (Pierce Biotechnology, Inc., Rockford, IL, USA) and the relative protein expression was analyzed using Image-Pro plus software (version 6.0; Media Cybernetics, Inc., Silver Spring, MD, USA), represented as the density ratio versus GAPDH.

### Transfection

Lipofectamine 2000 (Life Technologies) was used to perform cell transfection, according to the manufacturer’s instructions. For FSCN1 functional analysis, SW480 cells were transfected with FSCN1-specific small interfering (si)RNA or co-transfected with FSCN1 plasmid and miR-133a mimics. For miR-133a functional analysis, SW480 cells were transfected with scrambled miRNA as a negative control (NC), miR-133a mimics or miR-133a inhibitor (Life Technologies).

### Dual Luciferase reporter assay

A QuikChange II Site-Directed Mutagenesis kit (Agilent Technologies, Inc., La Jolla, CA, USA) was used to generate a mutant 3′-UTR of FSCN1, according to the manufacturer’s instructions. The wild-type or mutant 3′-UTRs of FSCN1 were inserted into psiCHECK™2 vectors (Promega Corporation, Madison, WI, USA) and the resultant psiCHECK™-2-FSCN1-3′-UTR and psiCHECK™-2-mutant FSCN1-3′-UTR vectors were transfected into SW480 cells, with or without 100 nM miR-133a mimics, respectively. The two groups of SW480 cells were incubated at 37°C with 5% CO_2_ for 48 h, followed by analysis of their luciferase activities using an LD400 luminometer (Beckman Coulter, Fullerton, CA, USA). Renilla luciferase activity was normalized to firefly luciferase activity.

### Invasion assay

Transwell assay (Corning, Inc., Corning, NY, USA) was performed to determine the cell invasive capacity. A cell suspension containing 5×10^5^ cells/ml was prepared in serum-free media for the wild-type and mutant-transfected SW480 cells. Next, 500μl DMEM supplemented with 10% FBS was added into the lower chamber, and 300μl cell suspension was added into the upper chamber. Subsequently, cells were incubated at 37°C with 5% CO_2_ for 24 h. Cells on the upper surface was removed using a cotton-tipped swab, while cells on the lower surface were stained for 30 min. Microscopy was use to count the cell number in at least five randomly selected fields.

### Statistical analysis

SPSS software (version 17.0; SPSS, Inc., Chicago, IL, USA) was used to perform statistical analyses. Differences were analyzed by performing one-way analysis of variance and all data were expressed as the mean ± standard deviation. P<0.05 was considered to indicate a statistically significant difference.

## Results

### miR-133a expression in colorectal cancer tissues and cells

The expression level of miR-133a was determined by performing RT-qPCR on colorectal cancer tissues and their paired normal adjacent tissues. As indicated in Fig. 1A, the expression level of miR-133a in colorectal cancer tissues was significantly decreased compared with the paired normal tissues (P=0.0004). In addition, miR-133a expression was examined in three colorectal cancer cell lines, including HT29, SW480 and SW620; it was identified that miR-133a was also downregulated in colorectal cancer cells compared with the normal intestinal epithelium cell line, NCM460 (P=0.0001, P<0.0001 and P=0.0001 vs. HT29, SW480 and SW620 cells, respectively) (Fig. 1B). SW480 cells demonstrated the most marked downregulation of miR-133a (Fig. 1B), thus, SW480 cells were used in the subsequent experiments.

### FSCN1 is a direct target of miR-133a

TargetScan software (http://www.targetscan.org/) was used to perform bioinformatic analysis, which demonstrated that the putative seed sequences for miR-133a at the 3′-UTR of FSCN1 were highly conserved. Thus, wild-type and mutant FSCN1 3′-UTRs were generated as indicated in Fig. 2A. A dual luciferase reporter assay was performed on the SW480 cells; notably, the luciferase activity was only significantly reduced in the SW480 cells co-transfected with the wild-type FSCN1 3′-UTR and miR-133a mimics (P=0.008; Fig. 2B), indicating that miR-133a directly targets the 3′-UTR of FSCN1 in SW480 cells.

### miR-133a regulation of FSCN1 protein expression levels

The role of miR-133a in the regulation of FSCN1 protein expression levels was additionally investigated in colorectal cancer SW480 cells. Following transfection of SW480 cells with scramble miRNA, miR-133a mimics or miR-133a inhibitor, the expression level of miR-133a in each group was detected to confirm that the transfection efficiency was satisfactory (Fig. 3A). After transfection with miR-133a mimics, the expression level of miR-133a was significantly increased when compared with the control group (P=0.0001). By contrast, after transfection with the miR-133a inhibitor, the expression level of miR-133a was significantly reduced when compared with the control group (P=0.005). Subsequently, the protein level of FSCN1 in each group was determined using western blotting. As indicated in Fig. 3B, upregulation of miR-133a induced a decrease in the protein expression levels of FSCN1 (P=0.0001), while downregulation of miR-133a resulted in upregulation of FSCN1 protein expression levels (P=0.008) in SW480 cells. Thus, the protein expression levels of FSCN1 appear to be negatively mediated by miR-133a in colorectal cancer SW480 cells.

### miR-133a suppresses colorectal cancer cell invasion via FSCN1 inhibition

The role of miR-133a and FSCN1 in the regulation of colorectal cancer cell invasion was additionally investigated by conducting an invasion assay. SW480 cells were transfected with miR-133a mimics or FSCN1-specific siRNA, or co-transfected with miR-133a mimics and FSCN1 plasmid. Upregulation of miR-133a and inhibition of FSCN1 significantly suppressed SW480 cell invasion (P=0.006 and P=0.0001, respectively); however, the inhibitory effect of miR-133a upregulation on SW480 cell invasion was notably reversed by overexpression of FSCN1 (Fig. 4). These findings indicate that miR-133a may inhibit SW480 cell invasion via direct inhibition of FSCN1.

## Discussion

The present study identified that the expression level of miR-133a was markedly decreased in colorectal cancer tissues and cells, when compared with paired adjacent tissues. However, FSCN1, a direct target of miR-133a, was markedly upregulated in colorectal cancer tissues. Furthermore, FSCN1 expression was negatively modulated by miR-133a at a post-transcriptional level in colorectal cancer cells. Thus, this investigation into the molecular mechanism of colorectal cancer cell invasion revealed that miR-133a may, at least partially, inhibit colorectal cancer cell invasion via FSCN1 inhibition.

It is well-established that the deregulation of miRNAs contributes to various types of human cancer (17). For example, the loss of miR-133a expression was associated with lymph node metastasis, high clinical stage and a shorter relapse-free survival period in breast cancer patients (18). In the present study, the expression level of miR-133a was remarkably reduced in colorectal cancer tissues compared with paired normal adjacent tissues. Furthermore, miR-133a was downregulated in colorectal cancer cell lines compared with normal intestinal epithelium NCM460 cells. This downregulation of miR-133a expression in colorectal cancer tissues has previously been reported; for example, Arndt *et al* (19), performed mirVana™ miRNA Bioarrays to examine the miR-133a expression profile in eight colorectal cancer cell lines, 45 human colorectal cancer samples of different stages and four paired normal colorectal tissue samples. It was identified that loss of miR-133a was associated with colorectal cancer progression. Additionally, Sarver *et al* (20) proposed that miR-133a was downregulated in colorectal cancer tissues and, recently, Dong *et al* (21) reported that miR-133a was notably downregulated in primary colorectal cancer tissues compared with paired adjacent normal tissues. Furthermore, ectopic expression of miR-133a significantly inhibited colorectal cancer cell growth *in vitro* and *in vivo*, possibly by inducing G0/G1-phase arrest. Thus, deregulation of miR-133a appears to be involved in the development and progression of colorectal cancer. However, the specific role of miR-133a in the regulation of colorectal cancer cell invasion remains unclear.

FSCN1 has been demonstrated to act as an oncogene, and its expression level was significantly upregulated in various types of cancer, including ovarian carcinoma (22), gastric cancer (23) and colorectal cancer (24). Furthermore, upregulation of FSCN1 was proposed as a mechanism of epithelial to mesenchymal progression in cancer, conferring specific invasive properties on cancer cells (25). Previously, the association between miR-133a and FSCN1 has been reported in a number of other cancers, including bladder cancer (26), breast cancer (18) and esophageal squamous cell carcinoma (27). For example, it was reported that miR-133a repressed the mRNA and protein expression of FSCN1 in bladder cancer (26), as well as targeting the expression of FSCN1, and suppressing tumor cell invasion and migration in breast cancer (18). Additionally, it was demonstrated that miR-133a acts as a key tumor-suppressive miRNA to directly inhibit the expression of FSCN1 in esophageal squamous cell carcinoma (27). However, the specific roles of miR-133a and FSCN1, as well as their association in colorectal cancer, remain to be investigated. The present study determined that miR-133a regulates the protein expression levels of FSCN1 by directly targeting the 3′-UTR of FSCN1 mRNA in colorectal cancer SW480 cells. By performing gain of function assays, miR-133a overexpression was identified to significantly inhibit cell invasion in colorectal cancer SW480 cells, similar to the effect of FSCN1 downregulation. Furthermore, FSCN1 overexpression reversed the inhibitory effect of miR-133a upregulation on SW480 cell invasion, clarifying that FSCN1 acts as a downstream effecter of miR-133a in SW480 cells.

In conclusion, miR-133a was identified to exhibit an at least partial inhibitory effect on colorectal cancer cell invasion via the suppression of FSCN1 protein expression, which was identified as a direct target of miR-133a. Thus, the present study proposes that FSCN1 may serve as a promising therapeutic target for colorectal cancer metastasis. Future research should focus on *in vivo* studies to further understand the role of the miR-133a/FSCN1 axis in colorectal cancer growth and metastasis.

## Figures and Tables

**Figure 1:** (A) RT-qPCR was performed to examine the relative expression of miR-133a in 17 CRC samples (cancer) and their paired normal samples (normal). ^*^P<0.01, vs. normal. (B) RT-qPCR was performed to examine the relative expression of miR-133a in human CRC lines (HT29, SW480 and SW620), as well as a normal intestinal epithelium cell line (NCM460). ^*^P<0.01, vs. NCM460. RT-qPCR, reverse transcription-quantitative polymerase chain reaction; CRC, colorectal cancer.

**Figure 2:** (A) The seed sequences of miR-133a against the wild-type or mutant 3′-UTR of FSCN1. (B) Luciferase reporter assay identified that co-transfection of SW480 cells with miR-133a mimics and wild-type FSCN1 3′-UTR caused a significant decrease in luciferase activity, whereas co-transfection with mutant FSCN1 3′-UTR and miR-133a mimics showed no significant difference compared with the control group. Control, cells co-transfected with blank vector and wild-type SP1R1 3′-UTR or mutant FSCN1 3′-UTR. ^*^P<0.01, vs. control. FSCN1, Fascin1; UTR, untranslated region; miR, microRNA; NC, negative control.

**Figure 3:** (A) Reverse transcription-quantitative polymerase chain reaction was performed to determine the relative expression level of miR-133a in SW480 cells transfected with scramble miRNA (NC), miR-133a mimics and miR-133a inhibitor. (B) Western blot analysis was performed to examine the protein expression level of FSCN1 in SW480 cells transfected with miR-133a mimics and miR-133a inhibitor. Control, SW480 cells with no transfection. ^*^P<0.01, vs. control. miR, micro RNA; NC, negative control; FSCN1, Fascin1.

**Figure 4:** Transwell assay determined the invasion capacity in SW480 cells transfected with miR-133a mimics or FSCN1 siRNA, or co-transfected with miR-133a mimics and FSCN1 plasmid. Control, SW480 cells with no transfection. ^*^P<0.01, vs. control. miR, micro RNA; FSCN1, Fascin1; siRNA, small interfering RNA.
